The article "Relationship between Acute Respiratory Tract Infection and the Serum 25(OH) D3 Level in Chronic Kidney Disease Patients and Its Prevention and Treatment" was retracted in 2023. Reasons: unreliable results or conclusions; concerns about the data; concerns about the peer review; concerns about the citations.

# Relationship between Acute Respiratory Tract Infection and the Serum 25(OH) D3 Level in Chronic Kidney Disease Patients and Its Prevention and Treatment

**DOI:** 10.1155/2022/2550686

**Published:** 2022-08-04

**Authors:** De-Han Cai, Jun Wang, Aimin Zhong, Xiao-Lin Fang

**Affiliations:** ^1^Nephrology Department in Jiangxi Provincial People's Hospital Affiliated to Nanchang Medical College, Nanchang 330006, Jiangxi, China; ^2^Department II of Respiratory and Critical Care in Jiangxi Provincial People's Hospital Affiliated to Nanchang Medical College, Nanchang 330006, Jiangxi, China

## Abstract

Observational studies and randomized controlled studies propose that vitamin D plays a significant role in preventing acute respiratory tract infection (RTI); however, results are inconsistent and the optimal serum 25-hydroxyvitamin D (25-OH-D3) concentration remains unknown. This study explores the risk factors associated with acute RTI in patients with chronic kidney disease (CKD) and analyzes its correlation with serum 25-OH-D3 levels, to provide appropriate preventive treatment measures for CKD patients complicated with acute RTI. Seventy cases of CKD patients treated in the department of nephrology of Jiangxi Provincial People's Hospital are recruited as the research objects and divided into a control group (CKD without RTI) and an observation group (CKD with RTI), with 35 cases in each group. The laboratory indexes and serum 25-OH-D3 levels are compared between the two groups. The area under the receiver operating characteristic curve (ROC) of 25-OH-D3 in the diagnosis of CKD patients complicated with RTI is 0.892, and the standard error is 0.038. The glomerular filtration rates (GFR) are 48.32 ± 9.87 mL/min and 50.18 ± 20.71 mL/min in the control group and the experimental group, respectively, with no statistical significance between the two groups (*P* > 0.05). The serum 25-OH-D3 content in the control group (35.08 ± 6.2 nmol/L) is dramatically higher than that in the observation group (20.71 ± 5.87 nmol/L) (*P* < 0.05). The proportion of patients with diabetes mellitus (DM) in the control group and observation group is 25.71% and 68.57%, respectively, with a considerable difference (*P* < 0.05). In the control group and the experimental group, the proportion of patients with oral vitamin D receptor agonists is 54.29% and 11.43%, respectively, and the difference is significant (*P* < 0.05). Results show that the serum 25-OH-D3 level is highly correlated with the occurrence of RTI in CKD patients. In addition, it is related to patients' age, DM, and vitamin D receptor agonists.

## 1. Introduction

Respiratory tract infection (RTI) is a common respiratory disease. Chronic kidney disease (CKD) often leads to patients' low immune function and weakened resistance, leading to the invasion of other pathogenic microorganisms such as viruses and bacteria, thus causing secondary infection such as RTI and further weakening patients' ability to resist diseases [1]. Therefore, this is also one of the reasons why kidney disease is difficult to cure, often leading to aggravation and recurrent attacks in patients who have recovered or are in the process of recovery [2]. Immune complex nephritis caused by antigen-antibody reaction aggravates the disease of patients and may even lead to renal failure in patients with renal insufficiency [3]. Therefore, for CKD patients, it is necessary to actively prevent colds and upper RTI, to effectively avoid the recurrence of kidney disease [4].

The article "Relationship between Acute Respiratory Tract Infection and the Serum 25(OH) D3 Level in Chronic Kidney Disease Patients and Its Prevention and Treatment" was retracted in 2023. Reasons: unreliable results or conclusions; concerns about the data; concerns about the peer review; concerns about the citations.

Studies found that the risk of infection in CKD patients is three to four times higher than that in normal people and the prevention of various infections in the upper respiratory tract and urinary tract can effectively reduce the risk of rapid deterioration of renal function in CKD and delay the progression of CKD [5]. 25-OH-D3 is a cholesterol derivative, which is a precursor of active cholesterol metabolites in the body and becomes biologically active after being transformed into 25-OH-D3 [6]. Vitamin D3 is absorbed and stored in plasma, liver, fat, and muscle and transferred to the liver by blood to be transformed into 25-OH-D3 and stored in the liver [7]. Once hydroxylated, vitamin D3 is more easily circulated in the blood due to increased water solubility due to the addition of a hydroxyl group and becomes the main circulation form in blood [8, 9]. The normal level of 25-OH-D3 in serum is between 30 and 100 ng/mL. If the level is less than 30 ng/mL, vitamin D deficiency is considered. Vitamin D deficiency is considered if its concentration is greater than 30 ng/mL and less than 50 ng/mL [10].

Several studies have explored the relationship between 25-OH-D3 serum concentration and RTI and the impact of vitamin D supplementation on RTI [11]. Two recent meta-analyses of observational studies found the relationship between 25-OH-D concentration and RTI incidence in children [12, 13]. The first analysis included the case-control studies in children with age < 5 years and reported higher odds of 25-OH-D shortage in those with RTI. The second found an opposite association between prenatal maternal 25-OH-D concentration and risk of RTI in the children. Furlong et al. [14] conducted 19 observational studies and found a significant inverse association between 25-OH-D concentration and risk of RTI. Jolliffe et al. [15] completed a systematic review of 25 observational studies and 14 randomised-controlled trials (RCTs) in 2013 and found an inverse relationship between 25-OH-D composition and risk of RTI. Respiratory infections are predominant in winter. Vitamin D such as 25-OH-D may play a vital role in the host's defense against RTI. Reports from epidemiological investigations have associated a deficiency of vitamin D to increased susceptibility to acute viral respiratory infections [16]. Numerous human and animal studies have proved a defensive role of high maternal serum levels of vitamin D in the case of viral infection, proposing that high vitamin D serum levels in pregnancy might protect the infant from developing RTI or viral-induced wheezing incidents. Camargo et al. [17] proposed that high cord blood 25-OH-D levels are related with a lower risk of RTI and childhood wheezing risk and severity and give a symptom of the optimal 25-OH-D density for acute RTI inhibition and management. The low serum 25 (OH) vitamin D level is related to viral RTI in 743 children (3–15 years old) in a study conducted between December 2008 and January 2009 [18].

The article "Relationship between Acute Respiratory Tract Infection and the Serum 25(OH) D3 Level in Chronic Kidney Disease Patients and Its Prevention and Treatment" was retracted in 2023. Reasons: unreliable results or conclusions; concerns about the data; concerns about the peer review; concerns about the citations.

Studies revealed that vitamin D deficiency is also associated with the occurrence and development of DM and vitamin D deficiency can increase the risk of cardiovascular adverse events such as hypertension, coronary heart disease, and cardiac insufficiency [19]. In recent years, the role of 25-OH-D3 in immune function regulation, renal protection, and cardiovascular protection has gradually attracted attention [20, 21]. This study examines the risk factors associated with acute RTI in patients with CKD and analyzes its correlation with serum 25-OH-D3 levels, to provide appropriate preventive treatment measures. Seventy cases of CKD patients are recruited as the research objects and divided into the control group and observation group, with 35 cases in each group. Results show that the serum 25-OH-D3 level is highly correlated with the occurrence of RTI in CKD patients. In addition, it is related to patients' age, DM, and vitamin D receptor agonists.

The rest of the manuscript is organized as follows: Section 2 is about the material and methods.  Section 3 provides a detailed illustration of the obtained results.  Section 4 is about the discussion, and the conclusion is presented in Section 5.

## 2. Materials and Methods

### 2.1. Research Object and Grouping

In this study, 70 CKD patients who were admitted to the department of nephrology of Jiangxi Provincial People's Hospital from January 2017 to November 2020 were recruited as the subjects, with no limitation on pathological types and stages. Among them, 37 were male patients and 33 were female patients, aged from 45 to 75 years. Patients were divided into a control group (CKD without RTI) and an observation group (CKD complicated with RTI), with 35 patients in each group. This trial had been approved by Jiangxi Provincial People's Hospital's Medical Ethics Committee. Patients and their families understood the study content and methods and agreed to sign corresponding informed consent forms.  Table 1 shows the stages and glomerular filtration rates of CKD patients.

The article "Relationship between Acute Respiratory Tract Infection and the Serum 25(OH) D3 Level in Chronic Kidney Disease Patients and Its Prevention and Treatment" was retracted in 2023. Reasons: unreliable results or conclusions; concerns about the data; concerns about the peer review; concerns about the citations.

In this study, different patients were included. The patient inclusion criteria were: patients with renal impairment, including pathological and imaging abnormalities or abnormal urine tests, with GFR persistently lower than 90 mL/min, and duration was more than 3 months were included. Similarly, the patients having fever symptoms and upper respiratory inflammatory symptoms such as in the nose, throat, or para-nasal sinus were also included in the study. Likewise, the patient had symptoms of cough, phlegm, and lung rales and patients who agreed and were willing to cooperate with the study and sample collection were also included.

The exclusion criteria were as follows: patients with other systemic diseases or serious infectious diseases, patients with incomplete clinical data and information, patients who had recently taken glucocorticoids and other drugs for treatment, and patients undergoing hemodialysis or kidney transplantation were excluded from the study.

### 2.2. The 25-OH-D3 Structure

Regarding the molecular structure, 25-OH-D3 is the addition of a hydroxyl group to the 25-position carbon atom of vitamin D3 [22–24]. However, this addition occurs in the body through a series of biochemical reactions, through the 25-hydroxylase hydroxylation in the mitochondria of liver cells, which then forms 25-hydroxyvitamin D3 [25].  Figure 1 shows the structural formula of 25-OH-D3.

### 2.3. Research Methods

In this study, a questionnaire survey method was employed. A patient information questionnaire was designed and developed to record the basic information of the patients, including age, sex, clinical symptoms, CKD stage, and laboratory examination. Routine chest X-ray examination of RTI was considered in both experimental and control groups. Before the X-ray examination, the patient was placed in the upright and lateral position according to the doctor's guidance. The chest should be placed on the plate, the head should be tilted back later, the lower jaw should be placed on the upper edge of the plate, and the hands should be placed between the waist. During the examination, with the doctor's instructions, the patients can take an appropriately deep breath and hold their breath. Venous blood was taken in the morning after ten hours of fasting and water restriction. Fasting blood routine, albumin, serum creatinine (Cr), blood urea nitrogen (BUN), serum calcium, and parathyroid hormone (PTH) were determined. Hemoglobin and parathyroid hormone were identified by photoelectric colorimetry, serum albumin was determined by chemiluminescence, and serum creatinine was determined by urea nitrogen enzymatic kinetics.

The article "Relationship between Acute Respiratory Tract Infection and the Serum 25(OH) D3 Level in Chronic Kidney Disease Patients and Its Prevention and Treatment" was retracted in 2023. Reasons: unreliable results or conclusions; concerns about the data; concerns about the peer review; concerns about the citations.

Serum 25-OH-D3 was determined by colloidal gold immunochromatography. After blood samples were collected from patients, anticoagulant was added to them and stored at 2–8°C. The samples were restored to room temperature before detection. The test paper was taken out of the 25-OH-D3 quantitative detection kit (Shanghai Jianglai Biotechnology Co. Ltd.), and the kit was placed on a clean horizontal table. The serum sample was diluted with sample buffer in the proportion of 1 : 10 (10 *μ*L sample mixed with 90 *μ*L dilution), and a 100 *μ*L diluted sample was added to the well and time. The reagent card of reaction time of 15 min was put into a colloidal gold immunochromatography analyzer (Wanhua Puman Biological Engineering Co. Ltd.), and the results must be read immediately after the reaction.

When the detection result indicated “>100 ng/mL”, it meant that 25-OH-D3 in the detected blood sample was higher than the upper limit of the detection range. At this point, if the accurate value was to be determined, the buffer was diluted again and the test was repeated. The sample concentration was the test value multiplied by the dilution factor. The determination of test results was shown in Table 2.

### 2.4. Observation Indicators

After venous blood was extracted from patients in the experimental and control groups, serum albumin, Cr, BUN, serum calcium, PTH, and serum 25-OH-D3 levels were determined. The correlation between the serum 25-OH-D3 content and RTI in CKD patients was examined by comparing the index difference between patients with RTI and patients without RTI.

### 2.5. Statistical Methods

SPSS 22.0 software [26] was employed for data analysis. Measurement data were presented as mean ± standard deviation ($\overset{¯}{x\pm s}$) and counting data as a percentage (%). Analysis of variance was adopted for pairwise comparison. *P* < 0.05 indicated that the difference was statistically significant.

## 3. Results

### 3.1. Preoperative Blood Indexes of Patients

RTI X chest radiographs can be used to determine the extent, distribution, and extent of the lesions [27], and an etiological examination was performed according to the X-ray findings. The common manifestations of RTIX radiography were pulmonary texture enhancement and small nodular shadows dominated by inflammatory congestion, edema, and exudative lesions of the bronchial wall, as well as patchy shadows and segmental and lobular consolidation caused by various causes of bronchopneumonia.  Figure 2 shows the chest X-ray images of six CKD patients with RTI complications. The infected lesions are mostly located in the middle and lower lung fields, near the hilum and lower lung fields. There are enhanced lung texture, blurred-edge, patchy, nodular density-increased shadow, about 5 mm in size, patchy shadow distributed along the bronchus, and unclear boundary. In addition, radiographs show focal patchy shadows, focal ground glass shadows, diffuse patchy shadows, or diffuse ground-glass shadows about 2 cm in size in the lung field.

The article "Relationship between Acute Respiratory Tract Infection and the Serum 25(OH) D3 Level in Chronic Kidney Disease Patients and Its Prevention and Treatment" was retracted in 2023. Reasons: unreliable results or conclusions; concerns about the data; concerns about the peer review; concerns about the citations.

### 3.2. Basic Patient Information

Table 3 shows the comparison results of basic information between the control and observation groups. It can be seen that there are no considerable differences in the proportion of males and females in the two groups (*P* > 0.05). There were 14 patients under 60 years old in the control group, accounting for 40%, and only 6 patients under 60 years old in the observation group, accounting for 17.14%. The average ages of patients in the two groups were 55.21 ± 7.21 and 64.33 ± 6.8 years old. Patients with DM in the two groups were diagnosed and recorded. Results show that there are 9 cases (25.72%) with DM in the control group and 24 cases (68.57%) with DM in the observation group.

### 3.3. Diagnosis of RTI in CKD Patients with 25-OH-D3

The serum 25-OH-D3 levels of CKD patients with and without RTI were determined by colloidal gold immunochromatography. Many different critical values were set for a continuous variable, and the corresponding sensitivity and specificity at each critical value were calculated. The curve is shown in Figure 3 with sensitivity as ordinate and 1-specificity as abscissa, namely, receiver operating characteristic curve (ROC). Sensitivity is the percentage of affected people who test positive for certain diagnostic methods, also known as true positivity. Specificity shows the percentage of disease-free individuals who were negative for a diagnostic test, also known as the true negative rate. The diagnostic ROC curve was drawn to evaluate the diagnostic value of 25-OH-D3 for CKD patients complicated with RTI. The calculated area under the ROC curve is 0.892, and the standard error is 0.038.

### 3.4. Comparison of Laboratory Indicators between the Two Groups

Venous blood was extracted from CKD patients with and without RTI. Photoelectric colorimetry, chemiluminescence, and enzyme kinetics were adopted to determine the contents of serum hemoglobin, albumin, Cr, BUN, calcium, phosphorus, and parathyroid hormone.  Figure 4 shows that the serum hemoglobin and albumin contents in the control group are 112.38 ± 9.87 g/L and 33.9 ± 1.35 g/L, respectively. Serum hemoglobin and albumin contents in the observation group are 109.83 ± 10.23 g/L) and 34.21 ± 1.28 g/L, respectively, with no notable difference (*P* > 0.05). In addition, there are no considerable differences (*P* > 0.05) in serum Cr, BUN, serum calcium, phosphorus, and parathyroid hormone contents between the two groups.

The article "Relationship between Acute Respiratory Tract Infection and the Serum 25(OH) D3 Level in Chronic Kidney Disease Patients and Its Prevention and Treatment" was retracted in 2023. Reasons: unreliable results or conclusions; concerns about the data; concerns about the peer review; concerns about the citations.

### 3.5. GFR and 25-OH-D3 Levels between the Two Groups

The glomerular filtration rate (GFR) was measured in the two groups, and the serum 25-OH-D3 content was determined by venous blood sampling.  Figure 5 shows that the GFR of patients in the control group and the experimental group are 48.32 ± 9.87 mL/min and 50.18 ± 20.71 mL/min, respectively, without a considerable difference, indicating no considerable difference in GFR between CKD patients complicated with RTI and patients without RTI (*P* > 0.05). The serum 25-OH-D3 content in the control group (35.08 ± 6.2 nmol/L) is dramatically superior to that in the observation group (20.71 ± 5.87 nmol/L) (*P* < 0.05). That is, the serum 25-OH-D3 content of CKD patients complicated with RTI is inferior to that of CKD patients without RTI.

### 3.6. Analysis and Determination of Risk Factors for RTI in Patients with CKD

To analyze the risk factors of RTI in CKD patients, their age, gender, DM, and oral vitamin D receptor agonist were compared between the two groups.  Table 4 shows that patients over 60 years old in the control group and the observation group account for 60% and 82.86%, respectively, and there is a statistical difference in the complication of RTI between the two groups. Thus, the age of CKD patients is correlated with RTI to some extent, and the older the patients are, the more likely that they were to develop RTI. Patients with DM in the control group and the observation group account for 25.71% and 68.57%, respectively, and the difference is great. Therefore, DM may be associated with RTI in CKD patients. In addition, the proportion of patients taking vitamin D receptor agonists orally in the control group and the experimental group is 54.29% and 11.43%, respectively, presenting a remarkable difference. Hence, oral vitamin D receptor agonists may be associated with RTI in CKD patients and vitamin D receptor agonists may resist the occurrence of RTI to some extent.

### 3.7. Effect of Using Vitamin D on Complicated RTI

Statistics analysis was made on vitamin D usage in the two groups, and the comparison results are shown in Table 5. Vitamin D uses in the control group, and the experimental group is notably different, which means that vitamin D use is correlated with RTI in CKD patients to a certain extent. Furthermore, taking vitamin D in CKD patients may prevent the occurrence of RTI to a certain extent, which may have a certain therapeutic effect on RTI in CKD patients.

The article "Relationship between Acute Respiratory Tract Infection and the Serum 25(OH) D3 Level in Chronic Kidney Disease Patients and Its Prevention and Treatment" was retracted in 2023. Reasons: unreliable results or conclusions; concerns about the data; concerns about the peer review; concerns about the citations.

## 4. Discussion

There are many types of kidney diseases, but the more common ones are glomerulonephritis and pyelonephritis. At present, the etiology and pathogenesis of most patients suffering from kidney diseases are not clear. However, in recent years, research by Moustakim et al. [28] found that some CKD patients often had an atypical history of RTI before onset or were prone to RTI during treatment. Upper RTI can be directly infected by bacteria or caused by a variety of viruses, and these bacteria and viruses also have a certain impact on the kidney, which may lead to kidney disease [29]. On the one hand, bacteria and viruses can invade kidney organization directly; on the other hand, bacteria and viruses can serve as antigens and cause immune complex sex nephritis. Zeng et al. [30] pointed out that in the cold epidemic season, haematuria or proteinuria appeared in some CKD patients when their condition was relatively stable, mainly because there is an immune complex in the glomerulus calm, and cause damage to renal small vessels and capillaries, resulting in enhanced permeability. In addition, the upper RTI can not only cause kidney disease but also aggravate the disease of patients with kidney disease. For patients with renal insufficiency, it can also lead to kidney failure and heart failure. Uwaezuoke et al. [31] found that the risk of infection in CKD patients is three to four times higher than that in normal people. Prevention and treatment of infection can effectively reduce the risk of rapid deterioration of renal function in CKD and delay the progression of CKD. Therefore, timely and active prevention of respiratory tract and urinary tract infection in CKD patients plays a critical role in the pathogenesis, progression, and prognosis of kidney disease.

In this study, chest X-ray examination of CKD patients complicated with RTI showed that the common manifestations of RTIX radiography were pulmonary texture enhancement and small nodular shadows dominated by inflammatory congestion, edema, and exudative lesions of the bronchial wall, as well as patchy shadows and segmental and lobular consolidation caused by various causes of bronchopneumonia. The venous blood samples of RTI and uninfected patients were extracted to detect the laboratory indexes. It was found that there was no statistical significance in the contents of serum hemoglobin, albumin, Cr, BUN, serum calcium, phosphorus, and parathyroid hormone in CKD patients complicated with RTI (*P* > 0.05). The serum 25-OH-D3 content in the control group was dramatically superior to that in the observation group (*P* < 0.05), suggesting that the serum 25-OH-D3 content in CKD patients complicated with RTI was inferior to that in CKD patients without RTI. Similar to the finding of Meraz-Muñoz and García-Juárez [32], vitamin D deficiency was found to be associated with increased cardiovascular disease and mineral and bone metabolism disorders in CKD patients. Vitamin D is a fat-soluble steroid derivative, mainly derived from vitamin D3 and vitamin D2 ingested through food. Vitamin D forms 25-OH-D3 through the action of 25-hydroxylase and generates the active form of 1,25-hydroxyvitamin D3, exerting biological effects, and the kidney is the basic target organ of vitamin D. In addition, the analysis of related influencing factors found that the age of CKD patients, DM, and vitamin D receptor agonist had a certain correlation with RTI. The older the patients were, the more likely that they were to develop RTI, and vitamin D receptor agonists may resist the occurrence of RTI to some extent. Similar to the results of Rysz et al. [33], vitamin D may prevent the occurrence of RTI to a certain extent and may develop a certain therapeutic effect on RTI in CKD patients.

The article "Relationship between Acute Respiratory Tract Infection and the Serum 25(OH) D3 Level in Chronic Kidney Disease Patients and Its Prevention and Treatment" was retracted in 2023. Reasons: unreliable results or conclusions; concerns about the data; concerns about the peer review; concerns about the citations.

## 5. Conclusion

Respiratory tract infection (RTI) is a common respiratory disease Patients with CKD often have a reduced immune system and resistance, which allows other pathogenic microorganisms such as viruses and bacteria to infiltrate the body, resulting in secondary infections such as RTI and further compromising patients' ability to fight diseases. In this study, CKD patients were investigated to explore the risk factors associated with acute RTI in patients with CKD and analyze its correlation with serum 25-OH-D3 levels, to provide appropriate preventive treatment measures. The patients were rolled into a control group and an observation group according to whether they had RTI. The differences in laboratory indicators and serum 25-OH-D3 content between the two groups were compared to study the correlation between the two groups and the prevention of RTI. The results showed that serum 25-OH-D3 level was highly correlated with the occurrence of RTI in CKD patients. In addition, the occurrence of RTI was related to patients' age, DM, and vitamin D receptor agonists. Taking vitamin D had certain preventive and therapeutic effects on its infection. However, only the indexes of patients with or without the concurrence of RTI were compared, which had certain limitations. Moreover, few RTI-related factors were included, which may have a certain influence on the final evaluation indexes, thus affecting the accuracy and reliability of the study. Therefore, this aspect needs to be optimized and improved in the follow-up study, to conduct further research.

The article "Relationship between Acute Respiratory Tract Infection and the Serum 25(OH) D3 Level in Chronic Kidney Disease Patients and Its Prevention and Treatment" was retracted in 2023. Reasons: unreliable results or conclusions; concerns about the data; concerns about the peer review; concerns about the citations.

## Figures and Tables

**Figure 1:** 25-OH-D3 structural formula.

**Figure 2:** Chest X-ray images of the patients. (a–f) Represented six CKD patients complicated with RTI.

**Figure 3:** ROC curve of 25-OH-D3 for the diagnosis of RTI in CKD patients.

**Figure 4:** Comparison of laboratory indicators between the two groups. (a) Comparison of hemoglobin and albumin contents; (b) comparison of Cr and BUN; (c) comparison of serum calcium and phosphorus; (d) comparison of calcium-phosphorus product and parathyroid hormone content.

**Figure 5:** Comparison of GFR and 25-OH-D3 content between the two groups. ^∗^Statistically considerable difference versus the control group (*P* < 0.05).

**Table 1:** Staging of CKD.

CKD stage	Glomerular filtration rate (GFR) (mL/min)	Blood phosphorus (mmol/L)
1	>90	/
2	60–89	/
3	30–59	0.81–1.45
4	15–29	0.81–1.45
5	<15	1.13–1.78

**Table 2:** Determination of 25-OH-D3 detection results.

Display results (ng/mL)	Determination of results
>100	25-OH-D3 was higher than the upper limit of the detection range
30~80	25-OH-D3 was sufficient in the sample
10~30	25-OH-D3 was insufficient in the samples
<10	25-OH-D3 was absent in the samples

**Table 3:** Basic information of patients in the two groups.

Item	Type	Proportion (%)	
		Control group	Observation group
Gender	Male	17 (48.57%)	16 (45.71%)
	Female	18 (51.43%)	19 (54.29%)
Age	45~60	14 (40%)	6 (17.14%)
	60~70	12 (34.29%)	17 (48.57%)
	>70	9 (25.71%)	12 (34.29%)
DM	Yes	9 (25.71%)	24 (68.57%)
	No	26 (74.29%)	11 (31.43%)

**Table 4:** Risk factors analysis of CKD patients complicated with RTI.

Item	Type	Group		*P*	95% CI
		Control	Observation		
Age (years old)	<60	14 (40%)	6 (17.14%)	0.031	(1.028, 2.403)
	≥60	21 (60%)	29 (82.86%)		
Complicated with DM	Yes	9 (25.71%)	24 (68.57%)	0.018	(1.056, 2.576)
	No	26 (74.29%)	11 (31.43%)		
Gender	Male	17 (48.57%)	16 (45.71%)	0.586	(1.015, 2.038)
	Female	18 (51.43%)	19 (54.29%)		
Oral vitamin D receptor agonists	Yes	19 (54.29%)	4 (11.43%)	≤0.001	(1.138, 2.761)
	No	16 (45.71%)	31 (88.57%)		

**Table 5:** Effect of vitamin D on concurrent RTI.

Item	Type	Group		*P*
		Control	Observation	
Oral vitamin D intake	Yes	18	5	≤0.001
	No	17	30	

## Data Availability

The data that support the findings of this study are available from the corresponding author upon request.
